The article "Synthetic Epileptic Brain Activities with TripleGAN" was published in 2022. Journal: Comput Math Methods Med.

# Synthetic Epileptic Brain Activities with TripleGAN

**DOI:** 10.1155/2022/2841228

**Published:** 2022-08-27

**Authors:** Meiyan Xu, Jiao Jie, Wangliang Zhou, Hefang Zhou, Shunshan Jin

**Affiliations:** ^1^Minnan Normal University, China; ^2^OYMotion Technologies Co., Ltd., China; ^3^Beidahuang Industry Group General Hospital, China

## Abstract

Epilepsy is a chronic noninfectious disease caused by sudden abnormal discharge of brain neurons, which leads to intermittent brain dysfunction. It is also one of the most common neurological diseases in the world. The automatic detection of epilepsy based on electroencephalogram through machine learning, correlation analysis, and temporal-frequency analysis plays an important role in epilepsy early warning and automatic recognition. In this study, we propose a method to realize EEG epilepsy recognition by means of triple genetic antagonism network (GAN). TripleGAN is used for EEG temporal domain, frequency domain, and temporal-frequency domain, respectively. The experiment was conducted through CHB-MIT datasets, which operated at the latest level in the same industry in the world. In the CHB-MIT dataset, the classification accuracy, sensitivity, and specificity exceeded 1.19%, 1.36%, and 0.27%, respectively. The crossobject ratio exceeded 0.53%, 2.2%, and 0.37%, respectively. It shows that the established deep learning model of TripleGAN has a good effect on EEG epilepsy classification through simulation and classification optimization of real signals.

## 1. Introduction

Epilepsy is a chronic disease in which the sudden abnormal discharge of brain neurons leads to transient brain dysfunction. At present, there are about 50million epilepsy patients in the world. In all epilepsy patients, about 2/3 of the patients can control seizures through anticonvulsant drugs, 8-10% of the patients can control seizures through surgical resection of the focus, and another 25% of the patients cannot get effective treatment at present [1]. Timely and accurate detection of epilepsy plays an important role in the use of antiepileptic drugs; so, it is of great significance to design automatic detection methods for epilepsy. Epileptic EEG signal analysis technology involves interdisciplinary knowledge such as neuroscience, information science, and medicine. Many scholars have studied epileptic EEG from different perspectives. Common researches include epilepsy feature extraction and classification [2, 3], epilepsy prediction [4, 5], and focus localization [6, 7]. In the analysis of epileptic EEG, people hope that the computer can automatically find the distribution of EEG characteristics from a large number of EEG samples.

Typical methods for epilepsy feature extraction include cumulative energy [8], correlation dimension [9], spectral energy [10], and maximum Lyapunov exponent [11] and then use pattern recognition methods such as support vector machine and decision tree to classify EEG patterns over a period of time. Great progress has been made in the field of artificial neural networks [12]. The traditional feature extraction in image recognition has been replaced by the features learned by end-to-end neural networks, while the relevant research on epileptic EEG prediction still focuses on feature extraction and traditional pattern recognition methods [2, 13]. However, most traditional methods extract information from single channel or between two channels, ignoring the implicit spatial-temporal relationship between multiple channels, and lack of extraction of epileptic EEG synchronous pattern change features.

The prediction of epileptic seizures has always been one of the hot issues in clinical research. In clinical diagnosis, doctors often take spike wave, sharp wave, spike slow complex wave, and other paroxysmal EEG abnormalities as the characteristics of epileptic signals [14]. Some clinical studies have shown that some precursors that predict seizures can be found before seizures [14]. Epilepsy is a process in which epileptic foci cause excessive synchronous discharge of other neurons. Therefore, the abnormal synchronous pattern reflects the evolution of epilepsy. Many clinical studies have found that there are differences in synchronization and desynchronization patterns between preseizure and interictal periods [15]. It is very important to study the diffusion law of abnormal discharge activity in the brain for the prediction of epilepsy.

EEG source localization is the problem of estimating the source of EEG activity from a given scalp EEG distribution, which is usually called the inverse problem of EEG. At present, the methods used to locate EEG activity sources mainly include equivalent current dipole (ECD) [16], sparse and Bayesian framework [17], beamforming and scanning algorithms [18], minimize L2 normal family [19], and nonlinear post hoc normalization [20]. In recent years, more researches have been made on introducing the timing pattern of the signal in the process of determining the position of the source signal [16–18]. After introducing the time information, the adjacent temporal signals can provide more observation data for the underdetermined EEG inverse problem, thus compressing the solution space and making the inverse problem easier to solve. On the other hand, the temporal pattern of EEG signals also plays an important role in the reconstruction of source activity. Based on the above analysis, this work extracts recognition features from the correlation between the amplitude of scalp EEG signals and the location of EEG signals caused by epileptic lesions and conducts in-depth learning of EEG epilepsy based on the dual GAN model. The main innovations and contributions are as follows:

- According to the local signal characteristics of epileptic EEG such as spike wave, sharp wave, and spike slow complex wave, the local virtual representation of epileptic EEG signal is studied. This paper proposes that GAN machine learning approach the real data to improve the robustness of data recognition
- The local feature enhancement of EEG signals can effectively solve the expression of epileptic EEG feature clustering and make the feature clustering of EEG signals more accurate
- GAN is used to perform arithmetic operation in the potential space (vector space) to convert the EEG clustering features into operations in the corresponding feature space. The generated data is no different from the real samples. Finally, the discriminator cannot correctly distinguish the generated data from the real data, so as to obtain more strengthened classification features

In a word, this paper puts forward new ideas on feature clustering, reinforcement and end-to-end classification, and recognition of epileptic EEG, which provides a new tool for automatic diagnosis.

## 2. Method

### 2.1. EEG Epilepsy Signal Generator

The generative countermeasure network (GAN) is mainly used to generate images. Great progress has been made in the stability and quality of generated images through different regularization methods [21, 22] and gradually increasing image resolution in training [23]. However, there are not many researches on time series. [24] designed temporal-spatial-frequency with mean-squared-error (TSF-MSE-based) loss function that reconstructs signals by computing the MSE from time-series features, common spatial pattern features, and power spectral density features.

In this study, parameters were migrated from the original signal, and the required source activation was repeated many times to generate a simulated model of EEG epilepsy. Firstly, the samples of source data are randomly selected as the initial epilepsy prediction samples, and a set of time series datasets with 4 s temporal window are quickly generated by using seed-g toolbox. Then, the TripleGAN model is used to selectively fine-tune the input-output paired in the target dataset to make it approach the real target.

### 2.2. Clustering Feature Extraction Methods

In the analysis and processing of epileptic EEG signals, there are many unsupervised dimensionality reduction feature extraction methods, such as model of PCA [25], ICA [26], and AR [27]. The method of unsupervised clustering is to mine the characteristics of samples according to the distribution of samples from the perspective of data-driven. Clustering models are mainly divided into partition-based clustering, density-based clustering, and signal self-coding-based clustering [28]. The clustering algorithm of EEG signals can mine the distribution rules between time series samples and find key sample patterns. Although the features extracted by the clustering algorithm cannot correspond to clear physical meaning, they can be used as a key component in feature extraction and play an important role in many EEG studies [29].

This paper extracts features from three dimensions: temporal, frequency, and temporal-frequency.

The specific methods are as follows:

- Temporal feature is the most basic feature in EEG signal processing, which is extracted by directly observing and calculating the original signal. We use a previous achievement [30] for the extracting the temporal model, see Figure 1
- The frequency domain feature is filtered by the method, which can distinguish the obvious change of EEG energy during seizures, see Equation (1)

(1) $$\begin{array}{c} P\left(\omega \right)=\overset{+\infty }{\underset{-\infty }{\sum }}r\left(k\right)e^{-i\omega k}. \end{array}$$

Wavelet analysis is used in the temporal-frequency domain to transform the one-dimensional signal in the temporal into the two-dimensional space of one scale in the temporal, and the frequency bands are divided at multiple levels for more precise feature decomposition, see Equation (2), which Ψ^∗^(*n* − *b*/*a*) is the conjugate function of Ψ(*n* − *b*/*a*).

(2) $$\begin{array}{c} W_{\Psi }=f\left(n\right),\Psi =\left(\frac{n-b}{a}\right)=\frac{1}{\sqrt{a}}\underset{n}{\sum }\Psi^{*}\left(\frac{n-b}{a}\right). \end{array}$$

Each of the three characteristics perform its own duties. In particular, wavelet packet analysis further decomposes the high-frequency part of multiresolution analysis that is not subdivided, and it has the excellent property of further dividing and thinning the spectrum window that widens with the increase of scale. Therefore, it has better temporal-frequency characteristics and improves the accuracy of EEG signal analysis [31].

### 2.3. TripleGAN Model

Inspired by the dual learning of natural language translation [31], we have developed a novel TripleGAN mechanism. DualGAN [32] trains the image converter with two sets of unlabeled images from two domains. In the experiment of this paper, the original GAN learns the characteristics of EEG from the three dimensions of temporal, frequency domain, and FFT temporal-frequency domain, carries out closed-loop training of original signals and analog generated signals, and allows EEG features from any domain to be translated and then reconstructed, see Figure 2. Therefore, the recognition weight can be reasonably constructed from the three-dimensional features of EEG epilepsy recognition to improve the recognition performance.

In the process of learning, the optimization goal of the generation model is to generate fake EEG epilepsy data as much as possible, so as to obtain the statistical distribution law of the real data. The discriminant model is used to judge whether the given input data comes from the real data or the generated model. Finally, when a discriminant model cannot accurately distinguish whether the data generated by the generated model is forged, we think that both the discriminant model and the generated model have been raised to a higher level, and the data generated by the generated model is enough to imitate the data in the real world.

## 3. Experiments and Results

### 3.1. Experimental Setup

This paper implements the proposed framework consisting of TripleGAN and three feature methods and stacked EEG epilepsy emulation using Keras 2.4.3 machine learning. We used a machine equipped with 12th Gen Intel(R) Core(TM) i9-12900K CPU@3.20GHz, 32GB RAM, 1 TB HDD, and GeForce RTX 3090 GPU under 64-bit Ubuntu operating system for conducting experiments for solving classification problems as described in Tables 1 and 2 using an open EEG epilepsy dataset of CHB-MIT.

### 3.2. Dataset

CHB-MIT dataset [33] is jointly recorded by Boston Children's Hospital and Massachusetts Institute of Technology. It uses 10-20 international standard lead system to place electrodes, and 16 bit analog-to-digital converter samples the input signal at 256 Hz. It trained on 2 or more seizures per patient and tested on 916 hours of continuous EEG from 24 patients.

### 3.3. Experiment Results

For a fair comparison, this paper his model is further compared with state-of-the-art and baseline models to show its superior performance.

For subject-dependent classification, the proposed model is compared with the recently published Bi-GRU [34], which proposed bidirectional gated recurrent unit (Bi-GRU) neural network to facilitate the diagnosis and treatment of epilepsy. A comparison with the DLEK-GP [35] method adopts the classic common spatial pattern (CSP) and discriminative log-Euclidean kernel-based Gaussian process for distinguishing epileptic EEG signals. A further comparison with the EEGWaveNet [36] approach utilizes trainable depth-wise convolutions as discriminative filters to simultaneously gather features from each EEG channel and separate the signal into multiscale resolution. Lastly, the proposed CE-stSENet [37] proposes channel-embedding spectral-temporal squeeze-and-excitation network which can capture hierarchical multidomain representations in a unified manner with a variant of squeeze-and-excitation block. In Table 1, the TripleGAN outperforms the comparison approaches by 1.19 percentage points regarding mean accuracy, 1.36 percentage points regarding mean sensitivity, and 0.27 percentage points regarding mean specificity.

For subject-independent classification, also use EEGWaveNet [36] as one of the base line methods. A representative method with the sparse representation-based epileptic seizure classification based on the dictionary learning with the homotopy (DLWH) algorithm is proposed [38]. GDL [39] introduces deep learning-based epileptic seizure prediction models using electroencephalograms (EEGs) that can anticipate an epileptic seizure by differentiating between the preictal and interictal stages of the subject's brain. Finally, a forward-looking approach of LRCN [40] construct an 18-layer long-term recurrent convolutional network (LRCN) to automatic epileptogenic zone recognition and localization on scalp EEG. [41] implemented the real-time seizure detection using DB16-DWT in seven eigenvalues with the RUSBoosted tree Ensemble method. In Table 2, the TripleGAN outperforms the comparison approaches by 0.53 percentage points regarding mean accuracy, 2.2 percentage points regarding mean sensitivity, and 0.37 percentage points regarding mean specificity.

## 4. Discussion

This paper naturally extends GAN to TripleGAN to extract EEG information on three domains about temporal, frequency domain, and temporal-frequency and ensures that the distribution of EEG epilepsy features characterized by classifiers and generators converges to the data distribution. As a unified model, TripleGAN can simultaneously obtain the latest classification results in the in-depth generation model. In order to jointly to estimate these conditional distributions characterized by classifier networks and classification condition generator networks, this paper defines a joint discriminator network, whose only function is to distinguish whether the samples are from the real data distribution or from the model. In addition, in order to clarify the generation rules of EEG epileptic focuses, this paper smoothly transfers the input into three dimensional spaces and uses the sequential optimization of GAN network to generate data simulation. Next, we will conduct in-depth research on this part.

## 5. Conclusion

This paper proved that the artificial EEG signals are generated by the generative countermeasure network. This paper trains GAN step by step to generate artificial signals in a stable way, and the signals are very similar to single channel real EEG signals in temporal and frequency domain.

## Figures and Tables

**Figure 1:** Temporal feature extraction structure of each layer.

**Figure 2:** TripleGAN model structure.

**Table 1:** The subject-dependent comparison with the state-of-art methods for CHB-MIT dataset.

Criterion	Comparison method				TripleGAN
	Bi-GRU [34]	DLEK-GP [35]	EEGWaveNet [36]	CE-stSENet [37]	
Accuracy	98.49	97.42	98.39 ± 2.39	95.96	99.68 ± 0.32
Sensitivity	93.89	97.57	68.94 ± 21.12	92.41	98.93 ± 1.07
Specificity	98.49	97.26	99.25 ± 0.85	96.05	99.52 ± 0.48

**Table 2:** The subject-independent comparison with the state-of-art methods for CHB-MIT dataset.

Criterion	Comparison method					TripleGAN
	DLWH [38]	GDL [39]	EEGWaveNet [36]	LRCN [40]	DB16-DWT [41]	
Accuracy	95.06	95.38 ± 0.23	96.17 ± 2.95	99.00	96.38	99.53 ± 0.47
Sensitivity	95.06	94.47 ± 0.11	56.83 ± 24.44	84.00	96.15	97.26 ± 2.47
Specificity	95.06	94.16 ± 0.16	96.97 ± 3.13	99.00	96.76	99.37 ± 0.23

## Data Availability

The datasets during the current study are available from the corresponding authors on reasonable request.
